# The Effect of Standing Mats on Biomechanical Characteristics of Lower Limbs and Perceived Exertion for Healthy Individuals during Prolonged Standing

**DOI:** 10.1155/2022/8132402

**Published:** 2022-07-30

**Authors:** Yan Zhang, Yining Xu, Zixiang Gao, Hongjun Yan, Jianshe Li, Yichen Lu

**Affiliations:** ^1^Research Academy of Grand Health, Ningbo University, Ningbo 315211, China; ^2^Faculty of Sports Science, Ningbo University, Ningbo 315211, China; ^3^Faculty of Engineering, University of Pannonia, Veszprém 8200, Hungary; ^4^Ningbo Bohan Crafts Co., Ltd., Ningbo 315336, China; ^5^Department of Sport and Physical Education, Zhejiang Pharmaceutical College, Ningbo 315100, China

## Abstract

**Objective:**

To identify the effect of standing mats on biomechanical characteristics of lower limbs and perceived exertion for healthy adult individuals during a prolonged standing task.

**Methods:**

32 healthy college students were recruited in the randomized and cross-over designed trial according to the effect size and statistical power. After collecting the anthropometric data, each participant was asked to finish 2 sessions of 4-hour prolonged standing tasks on standing mats (MS) and hard ground (GS) in a random order and with a 72-hour interval rest. The plantar pressure distribution, foot morphology, and scores of the BESS (balance error scoring system) would be recorded pre- and posteach task. The Borg Rating of Perceived Exertion (RPE) would be collected during the whole task. Paired-samples *t* test was adopted to analyse the before and after difference within group and independent-samples *t* test was adopted to analyse the difference between groups separately.

**Results:**

(1) A prolonged standing task on both MS and GS have a negative effect on RPE and balance performance. (2) The negative effect on RPE and balance performance induced by MS is significantly smaller than that induced by GS. (3) Compared to GS, prolonged standing on MS has a lower peak plantar pressure and an implicit decrease in navicular drop and AHI (arch index).

**Conclusion:**

Standing mat tends to alleviate the fatigue induced by prolonged standing in lower limbs, optimize the distribution of plantar pressure, and maintain the stability.

## 1. Introduction

Standing is one of the basic human postures, in which an individual's trunk keeps straight with his or her bodyweight loaded by feet. During standing, the ankles should play the role of anchor points, by this way, the center of body weight would slightly swing in the sagittal plane in a motion pattern similar to an inverted pendulum and keep relatively still with the space static references [1]. Standing, which could be learned during 8 to 12 months old, is an easy to learn task [2]. Generally, standing causes few healthy threatens; however, there would be a risk of falling if someone cannot keep balance while standing. Besides, the posture of standing is also associated with some pathological symptoms. For example, a sudden change from a low center of gravity to a standing posture might be associated with postural hypotension, and prolonged standing could induce foot pain [3], leg stiffness [4, 5], low back pain [6, 7], and other complications [8].

Prolonged standing is common in many occupations such as workers in assembly lines, equipment operators, cashiers, teachers, greeters, and soldiers. Although the numbers are limited, previous studies have shown that prolonged standing would increase the risk of musculoskeletal disorders and cardiovascular diseases [9–12]. However, most of these previous studies were conducted in the working circumstances [13] and have not reached a consensus about the duration threshold of prolonged standing. Some previous studies claimed that a standing task for just 30 minutes could affect postural control and proprioception of the human body [14]. Moreover, a systematic review included 25 relative studies that explored the relationship between prolonged standing, and the symptoms in the low back and lower limbs showed that there was consistent evidence verifying the correlation between prolonged standing and low back symptoms, trunk flexion, and lumbar curvature, indicating that after a 71-minute prolonged standing task, lower back symptoms would reach clinically relevant levels, and for individuals who already had low back pain, the threshold was reduced to 42 minutes. This review recommended not standing for longer than 40 minutes to avoid musculoskeletal symptoms [15].

Previous studies mostly focused on the physical discomfort and physiological changes in the cardiovascular and musculoskeletal systems during prolonged standing [12, 16–20], and limited studies have explored the effects of prolonged standing on the biomechanics characteristics. The study attempted to investigate the mediating effect of joint mobility on the effect of prolonged standing on venous function suggesting that excessive joint mobility might be a risk factor for venous insufficiency, suggesting that it was necessary to assess joint mobility in individuals who should stand for a long-time during work [21]. Nelson-Wong and Callaghan explored the effect of prolonged standing from biomechanical perspectives that included the activation of trunk muscles, joint stiffness, and kinetic parameters, finding that subjects would develop low back pain during exposure to prolonged standing and show a decrease in rotational stiffness at lateral flexion, as well as an increase in center of pressure (COP) offset during the unilateral standing test after the exposure of prolonged standing. Moreover, the study also found that prolonged standing might result in a reduction in balance response and the ability to resist lateral loads on the trunk effectively [22]. The result was consistent with that of the study conducted by Duarte which demonstrated that there were three COP migration patterns during a task of unconstrained standing more than 30 minutes: (a) shifting, a fast-displacement of the average position of COP from one region to another; (b) fidgeting, a fast and large displacement and returning of COP to approximately the same position; and (c) drifting, a slow continuous displacement of the average position of COP [23].

According to the negative effect induced by prolonged standing, some countries have identified prolonged standing as a major ergonomic problem and have been seeking interventions [24]. At present, some interventions come from several different perspectives, for example, a previous study that compared the biomechanical and subjective response induced by prolonged standing on inclined surfaces of ±16°, stating that inclined standing surfaces could reduce subjective pain in individuals with lower back pain and should be recommended for use in occupational settings where prolonged standing was required [25]. Recently, a study compared the effects of wearing regular socks, compression socks which could create a pressure of 15 to 20 mmHg, and compression socks which could create a pressure of 20 to 30 mmHg on fatigue of calf muscles, edema of body segments, and discomfort in prolonged standing from a wearing-point perspective. This study found that compression socks appeared to be effective in reducing fatigue of calf muscles induced by prolonged standing, and the effect of 15-20 mmHg compression socks and 20-30 mmHg compression socks was similar [26]. Some researchers claimed that standing on a soft surface could reduce muscle fibre recruitment and tension and improve blood circulation, thus reducing musculoskeletal system discomfort and fatigue [27]. Madeleine's team examined the difference of physiological and biomechanical responses between prolonged standing in polyurethane pad surface (soft) and aluminum casting surface (hard), and the results showed, compared with prolonged standing on the soft surface, prolonged standing on a hard surface would make the calf sore and numb and increase the electromyographic signal of the soleus muscle and the displacement of the COP in the frontal plane. The study suggested that prolonged standing on a soft surface would be more comfortable and prevent the leg from feeling sore and numb [28].

After taking the cost-effectiveness in practical applications into consideration, there is limitation in offering adapts inclined standing surfaces for workers who are in exposure to prolonged standing. The limitation is not only from the heterogeneity of anthropometry and anatomy of human beings but also from that the quantification protocol of the best incline angle for different individuals has not been determined yet by the academy. Besides, considering the user's retention, it would be difficult to ask workers who should prolongedly stand to maintain uniform footwear in every workday.

Therefore, it seems that providing a soft standing surface for this kind of population has health promotion potential. At present, it is more common to provide special standing mats or insoles. Standing mats and insoles designed for prolonged standing individuals have the same mechanism, which is to achieve the purpose of optimizing the distribution of body mass by changing the material properties of the contact interface between the standing area and the plantar [29]. The properties of the standing surface material are important factors affecting the discomfort of prolonged standing [30]. The previous studies showed that absorption and transmission of ground reaction force during standing would be optimized, and the subjective comfort during prolonged standing would be improved when the material of the standing surface has greater elasticity, stiffness, and thickness [27]. A systematic review that published in 2018 demonstrated that there was moderate level of evidence supporting the use of cushioning materials for the reduction of perceived musculoskeletal discomfort of the lower limb and the lower back while standing at work, calling for larger, good quality prospective RCT intervention trials [31]. Most studies of the intervention for the adverse reactions caused by prolonged standing are aimed at the clinical population and workers of specific occupations, making it difficult to generalize their results to other populations. There are not enough studies on surface interventions on the change of biomechanical parameters and the subjective proprioception induced by fatigue after prolonged standing to provide guidelines or suggestions with a high level of evidence. Additionally, considering that since most workers, who are exposed in prolonged standing, have fixed workstations, it would be not only feasible but also convenient to provide standing mats at their workstations. Lastly, previous studies have not reached consensus on the significant positive effect of standing mat application on subjective fatigue, plantar pressure distribution, and individual's physical balance ability. The reason might come from the heterogeneity between study protocols such as the time of prolonged standing. This study was designed and conducted to explore the effects of a new-type polyurethane foamed standing mat on biomechanics characteristics of lower limbs and perceived exertion for young healthy individuals during a 4-hour prolonged standing task.

## 2. Materials and Methods

### 2.1. Participant Recruitment and Ethics

The recruitment information of volunteers would be published online by one of the researchers, and the volunteers would register their names and contact information. Necessary personal information such as name, age, gender, and basic health condition was collected and was screened according to inclusion and exclusion criteria for the trial by another researcher. In this period, all volunteers would not know anything about the trial. They would just know there was a prolonged standing task. Volunteers who met the inclusion criteria (participants) were randomly allocated by the second research group. In this period, all participants still did not know details about the trial. The inclusion criteria of participants were as follows: (1) from 18 to 60 years old; (2) free from endocrine, metabolic, neuromuscular, and musculoskeletal disorders; (3) BMI from 18.5 to 23.9 [32]; (4) without any diseases that are not clinically recommended for physical activity; (5) not engaged in any physical activity with moderate or above intensity for at least 6 months. The exclusion criteria of participants were as follows: (1) under 18 years old or over 60 years old; (2) with endocrine, metabolic, neuromuscular, or musculoskeletal disorders; (3) be clinically required not to participate in any physical exercise; (4) be asked to participate in the trial involuntarily; (5) participated in physical activity with moderate or above intensity within the last 6 months.

The software G∗Power (Version 3.1.9.3, Heinrich Heine University, German, https://www.psychologie.hhu.de/arbeitsgruppen/allgemeine-psychologie-und-arbeitspsychologie/gpower) was used to calculate the sample size. The two-tailed paired *t* test whose *α* error probability was set at 0.05, the effect size (*d*_*z*_) was set at 0.5, and the statistical power (1 − *β*) was set at 0.75. The *β* would be calculated by Equation (1), and the schematic diagram of the sampling distribution when the hypothesis is true and false was provided in Figure 1.

(1) $$\begin{array}{c} Z_{\beta }=\frac{\left(d-d_{\mu }\right)}{\sigma /\sqrt{n}}=\sqrt{n}\frac{d}{\sigma }-Z_{\alpha }. \end{array}$$

All participants had written informed consent, and the study was approved by the Institutional Ethics Committee of Ningbo University (ARGH20210804).

### 2.2. Study Protocol

The trial was randomized and cross-over controlled. Each participant was asked to finish two sessions of prolonged standing tasks, one of which was standing on a standing mat (MS, density: 200 D, hardness: 65-75, size: 1080 mm × 508 mm × 19 mm, Bohan Craft Co., LTD, Ningbo, China), and the other was standing on the hard ground surface (GS), which was a wooden floor. In both standing tasks, the participants were asked to stand barefoot.

Considering that previous studies discovered that significant subjective and physiological changes were not observed until a minimum of 3-hour exposure to standing and suggested longer testing durations [9, 31, 33] and the eight-hour system of labor in China society (usually 8 : 00 to 12 : 00 in the morning and 13 : 00 to 17 : 00 in the afternoon), in this trial, each prolonged standing task lasted 240 minutes. During the task, participants were asked to stand in front of a height-adjustable table (size: 1.0 m × 1.5 m) for daily office activities and were required not to use the table to support any body part except the forearm during the task. The participants were allowed to adjust the table to a comfortable height to support their forearms.

Each participant would have a 10 min rest after standing for 110 minutes and be allowed to walk or sit then perform the rest of the task which lasted 120 minutes. The participants were kept barefoot during the whole trial, and each participant was supervised by a researcher who was allowed to give verbal cues to ensure that every participant could complete the whole task according to the trial requirements. The schematic diagram of the trial and the photo of the testing site was presented in Figures 2 and 3. Since the aim of this study is to explore the effects of prolonged standing on standing mat and hard ground on biomechanical parameters and the physical balance ability of each participant, the difference within each group between pre and post a prolonged standing and the mean differences between groups would be calculated. To eliminate the interference of the learning effect, all the outcome measures would be taken pre and post each prolonged standing task.

### 2.3. Data Collection

#### 2.3.1. Perceived Exertion

The Borg Rating of Perceived Exertion (RPE), whose range of score was 6 to 15, was used to evaluate the perceived physical fatigue from the musculoskeletal system, of each participant. Each participant was asked to subjectively rate the overall physical fatigue of legs, the perceived standing surface hardness, and the discomfort of specific body areas (upper back, low back, hips, thighs, knees, calves, ankles, and planters) before and after prolonged standing on the hard ground and standing mat.

#### 2.3.2. Plantar Pressure Distribution

The Novel® Plantar Pressure Collecting System (Version PEDAR X, Novel, German) with 99 sensors was used to collect the plantar pressure distribution, the shift of COP, and the pressure between the touch-down area and different anatomical regions of the plantar. The calculation of the peak pressure in different anatomical regions of the plantar, arch index (AI), and the amplitude of COP was based on the zoning in the system according to the average geometric center offset of the area in which the plantar pressure reached the maximum value.

According to the zoning in the system, the whole touch-down area could be divided into hallux (BH), other toes (OT), medial foot (MF), lateral foot (LF), midfoot (M), and heel (H). The schematic diagram of the plantar zone divisions was provided in Figure 4. All sensors were individually calibrated before each test to reduce measurement system error.

#### 2.3.3. Balance Error Scoring System (BESS)

The BESS test was used to assess the physical stability of participants before and after prolonged standing on hard ground and a standing mat.

Each participant was asked to (1) stand on both feet: stand side by side on the test surface with the inside of the feet in contact, hands-on the anterior superior iliac ridge, eyes closed; (2) stand by single-foot: Stand on the test surface on the nondominant foot with hip flexion at about 30 degrees and knee flexion at about 45 degrees. Place both hands on the anterior superior iliac ridge with eyes closed; (3) stand on lunge posture: both feet should be placed on the test surface, the nondominant foot should be placed in the back, toes should be fully followed before contact, hands should be placed on the anterior superior iliac ridge, and eyes closed [34]. It should be emphasized that the BESS test is a wide-used standard physical balance test that could only represent an individual's physical ability to keep balance in different postures and could not represent the body's balance condition during the 4-hour prolonged standing task in this study.

Each test lasted 20 seconds, and the researchers recorded the number of turnovers. “Turnover” in the test was defined as (1) hands leaving the anterior superior iliac ridge, (2) open either eye, (3) tripping or falling, (4) abduction or flexion of the hip exceeds 30 degrees, (5) leave the test surface with either foot, and (6) leave the test surface for more than 5 seconds [35].

The final score was the total deduction score which was calculated after the BESS test was repeated 3 times.

#### 2.3.4. Plantar Morphology Assessment

AutoCAD software (Version 2018, Autodesk, USA) was used to assess the plantar morphological structure which included the instep height and ball of the foot length and calculate the arch height index (AHI), which equaled the ratio of the instep height and ball of the foot length.

### 2.4. Quality Control

The order of the two tests was randomized, and the SPSS Software 17.0 (SPSS, Inc., Chicago, IL, USA) was used for the allocation of the participants and generation of the randomized order. Moreover, to reduce the effect of biological circadian rhythm and the fatigue induced by the previous task, each task was arranged at the same time on the same day with a rest interval of 72 hours. Moreover, the assessment blinding was adopted in this trial, the researchers who supervised the participants during the task and those who collect the data were different, and the researchers responsible for collecting the data were not informed of the participants' allocation.

### 2.5. Statistical Analysis

The SPSS Software 17.0 (SPSS, Inc., Chicago, IL, USA) was used for statistical analyses. Paired-samples *t* test and independent-samples *t* test were adopted for within-group and between groups separately. Data would be presented as means and standard deviations except if otherwise specified and considered statistically significant at *P* < 0.05.

## 3. Results and Discussion

### 3.1. Sample Size and Participant Recruitment

The plot of the sample size and statistical power made by the G∗power software was presented in Figure 5. According to the plot and the calculated results, the trial should recruit at least 30 participants to guarantee a statistical power of more than 0.75. After considering the participants lost to follow-up and invalid data, the trial planned to recruit 36 subjects. Eventually, 36 students from Ningbo University were recruited, and after eliminating the invalid data, 32 participants completed the test. The anthropometric information of participants is shown in Table 1.

### 3.2. Perceived Exertion and Biomechanical Parameters

As shown in Figure 6(a) and Table 2, the Rating of Perceived Exertion (RPE) of feet, calves, knees, thighs, and lumbar was significantly increased after a prolonged standing task in both MS and GS. However, the RPE increase in MS was significantly smaller than that in GS (*P* < 0.05), especially around the lumbar area (*P* < 0.01), indicating that the intervention of a standing mat might effectively relieve the individual's fatigue caused by prolonged standing task and the fatigue in the low back area. Besides, it can be seen from Figure 6(b) and Table 2 that the amplitude of COP on the *x*-axis (*P* < 0.05) and *y*-axis (*P* < 0.05) in MS is significantly smaller than that of GS, indicating that the use of standing mat intervention might be able to maintain COP stability during prolonged standing. As was shown in Figure 6(c) and Table 2, the difference in peak plantar pressure was mainly concentrated in MF (*P* < 0.05), M (*P* < 0.05), and H (*P* < 0.05) areas, and those in MF, LF, M, and H in MS were all significantly smaller than GS. Moreover, the peak plantar pressure in the LF area decreased after prolonged standing tasks on both GS and MS whereas those in other plantar areas increased. These results showed that the standing mat might be able to reduce the pressure on the forefoot and heel effectively. In terms of AI, as shown in Table 2, in MS condition, AI increased and reached statistical significance, while that in GS almost did not change, indicating that the intervention of a standing mat might be able to support the arch of the foot and increase the touch-down area of the midfoot.

### 3.3. Balance Error Scoring System (BESS)

The results of the BESS balance test were shown in Figure 6(d) and Table 3. According to the results, the error score of the BESS test increased in both MS and GS after a prolonged standing task, suggesting that the body stability of participants decreases. However, in MS, the decreased instability of all test postures was significantly smaller than that in GS, indicating that the intervention of a standing mat might be able to reduce the degree or slow the rate of body stability decline.

### 3.4. Plantar Morphological Change

Morphological results of the foot scan were shown in Table 4. Regardless of prolonged standing in MS or GS, both the instep height and ball of the foot length were significantly decreased after a prolonged standing task (*P* < 0.05). In addition, the AHI was significantly decreased in GS (*P* < 0.05) but did not change significantly in MS (*P* > 0.05). Meanwhile, both in MS and GS, there was no statistically significant difference between groups in the instep height and ball of the foot length.

## 4. Discussion

The purpose of this study was to explore the effects of a new-type polyurethane foamed standing mat on biomechanics characteristics of lower limbs and perceived exertion for young healthy individuals during a prolonged standing task. The main findings were that prolonged standing, despite surface, standing mat, and hard ground lead to an increase in rating of perceived exertion and induce a negative effect on the individual's balance ability. However, the standing mat seemed to delay or reduce the increase of subjective discomfort in the lower limbs with a less negative effect on balance which reached a statistically significant difference between groups. Compared with prolonged standing on the hard ground, the COP amplitude, and the peak plantar pressure of the median foot, midfoot, and heel were lower during standing on a standing mat, and the instep height and ball of the foot length decreased less, and the AI changed less, which also reached statistical significance.

The increased RPE was consistent with the results of some previous studies. For example, a cross-sectional study published in 2012 found that prolonged standing was one of the major causes of psychological and muscle fatigue in production workers. In the study, participants who were exposed to prolonged standing for more than 5 hours every day were asked to fill out questionnaires that were used to assess psychological fatigue. Moreover, surface electromyography (sEMG) was used to assess muscle fatigue. Eventually, a moderate and positive correlation with a statistical significance between the changes in sEMG of erector spinae muscle and psychological fatigue was found according to the study's result [36]. Although the subjects in this study were all male, its result was consistent with this study, which might imply that there would be no gender difference in physical fatigue induced by prolonged standing and that it should be confirmed by further studies with female subjects. In terms of body balance ability, this study is the first to evaluate the effects of prolonged standing tasks on body balance ability on different standing surfaces in a young and healthy population. Previous studies have shown that prolonged standing tasks would reduce the adaptability of the posture control system in patients with Parkinson's disease or obesity [37], increasing the risk of falling [38]. This study also shows that prolonged standing tasks could also have a negative influence on the balance ability of young and healthy individuals with a potential mechanism that might be related to muscle fatigue. In addition, adults who are exposed to prolonged standing working circumstances would be at a higher clinical risk of low back pain and hip abductor muscle fatigue that include hip muscle and tensor fascia in daily life [39]. Furthermore, a study conducted by Marshall et al. in 2011 showed that a prolonged standing task of just 2 hours could make the gluteus medius muscle, which was one of the hip abductor muscle groups and plays an important role to maintain the stability of the pelvis and trunk, become fatigued, leading to a significant decrease in muscle strength and endurance [40]. However, the performance of balance is multifaceted and multidimensional, leading to the diversity and specificity of its assessment methods. Therefore, future research should explore the effects of prolonged standing tasks on various static and dynamic balance abilities and determine the specific influencing mechanism.

The results of the RPE assessment showed that the standing mat seemed to delay or reduce the increase of the subjective fatigue and discomfort of the lower limbs and reached a statistically significant difference between groups. The findings are consistent with those of some previous explorations that researched the effect of different contact surfaces on the prolonged standing subjective, physiological, and biomechanical parameters. Madeleine's team published a study in 1998, pointing out that, compared with a hard surface (aluminum casting surface), a soft surface (polyurethane surface) could decrease subjective discomfort of the lower body, alleviate leg swelling, weaker electrical signals in the calf triceps, and induce less fatigue after a prolonged standing task. Meanwhile, similar to this study, Madeleine's study also measured the amplitude and displacement of the COP in the sagittal plane and frontal plane and found that the amplitude and total angular displacement of the COP were larger in the process of standing on the hard surface for a long time, which was consistent with the results of this study [28]. At the same time, this study also found that the use of a standing mat had a less negative effect on balance which reached a statistically significant difference when compared with prolonged standing on hard ground. The possible mechanism of the positive effect induced by using a standing mat on RPE might come from the optimization of plantar pressure distribution. According to the change of peak plantar pressure in different foot areas, the peak plantar pressure changed less in all foot areas after prolonged standing tasks on a standing mat than on the hard ground, meaning that the functioning of the foot was maintained more. This phenomenon might be interpreted by the difference in muscle activation when standing on different surfaces. A similar phenomenon has been identified in a study conducted in 2021 with healthy computer workers as participants. This study found that standing mats were associated with reduced discomfort in lower-body and increased physical performance compared to the concrete floor after a 2-hour standing task and concluded that the use of standing mats showed potential to improve the ergonomic experience and lessen discomfort as well as accumulated musculoskeletal strain during prolonged standing [41].

In terms of intervention protocols that use a standing mat, Wiggermann's team compared the effects of 4 different types of standing mats and hard ground surfaces in 4-hour standing on ontological discomfort and bipedal center of COP deviation in 2013, finding that 3 of these 4 types of standing mats could reduce the discomfort after 4-hour standing with no significant difference compared with the control group. However, there were significant differences in the frequency of COP deviation within the three types of standing mats, and the COP deviation frequency was positively correlated with the degree of discomfort. Also, the study believed that the subjective report might be less sensitive for the intervention of standing mats, and the biomechanical parameters might have higher sensitivity and be a better choice of outcome measures [42]. In 2004, a study by Orlando's team investigated the fatigue and discomfort perceived by assembly line workers in different body segments after standing for 8 hours under three different standing conditions: ordinary floor, soft standing mat, and soft insole. It was found that general physical fatigue, leg fatigue, and discomfort were reduced by standing conditions with a standing mat and insole. Orlando's team found that there was a moderate positive correlation between the effect and variables such as age, height, body weight, and years of work. Their conclusion might be inferred according to the fact that older subjects and those with longer working lives reported less discomfort after standing with insoles, while subjects with less body height reported less discomfort when standing on ordinary floors and soft mats. At the same time, no statistically significant differences were found between RPE or discomfort in various parts of the body while standing on the ordinary floor. The results of Orlando's study could be considered consistent with those of this study since insole and standing mats have softer surfaces compared to the ordinary floor [27].

When it comes to intervention protocols that use a wearable device, Tarrade's team published a study that assessed the positive effect of custom foot orthoses for prolonged standing workers in 2019. The study assessed the participants' static balance and static and dynamic plantar pressure after a 3-week intervention protocol of using 3D printing custom foot orthoses and finally found that the subjects' subjective pain, discomfort, and leg stiffness were significantly reduced and the mean peak plantar pressure in static and dynamic posterior plantar area was significantly decreased after the intervention. Meanwhile, the mean peak plantar pressure in midfoot was significantly increased, and the balance between medial and lateral parts of the body was significantly improved. Therefore, the study suggested that custom foot orthotics could help the body balance the distribution of plantar pressure and provide better support and stimulation to the arch of the foot. The underlying mechanism might be that the orthotics transfer plantar pressure from the heel to the midfoot successfully [43]. Future studies should compare the effects of different intervention protocols on different populations with different standing duration.

Previous studies have not explored the morphological changes of the foot. This study is the first to assess the effects of prolonged standing on foot morphology using foot morphology scans with a result showed that after prolonged standing on a standing mat, there was less decline in the instep height and ball of the foot length, and less change in AHI, all of which were statistically significant. However, there was no statistically significant difference between the instep height and ball of the foot length, and there may be different hypotheses about the underlying mechanisms leading to this result, such as acute changes in the mechanical properties of plantar fascia or fatigue of the plantar intrinsic muscles, and the decrease of the ball of foot length might not mean a change on anatomical structure, since it seems that only long-term intervention has an effect on anatomical structure. Additionally, it cannot be ruled out that the precision of the assessment equipment or the sample size was insufficient, which leads to the inability to carry out statistical analysis of the results on a smaller spatial scale, which is also one of the limitations of this study. Moreover, as has been mentioned above, from the perspective of practical application, the use of pedals and external-used devices has some obvious limitations; therefore, the effect of pedals or external-used devices has not been taken into comparison in this study. It cannot be ruled out that the application of pedals and other devices would have better effects on RPE and biomechanical parameters during the prolonged standing task than a standing mat. Last but not the least, the standard deviation is greater than the mean value in some parameters, making the reliability of the results should be considered. Future studies should attempt to use more precise methods to monitor changes in foot morphology and musculoskeletal anatomy.

There are some limitations from a statistical perspective. On one hand, the hardness of the wooden floor (GS) was not tested before the trial, inducing the analysis of the difference between GS and MS partially qualitative, and the quantitative difference between standing grounds of different hardness is still unclear. On the other hand, the gender difference was not analyzed in this study. Considering that the stamina of prolonged standing within males and females might be different, further studies should balance the baseline difference in stamina.

## 5. Conclusions

In conclusion, the results of this study support the fact that the utilization of a standing mat alleviates perceived exertion of lower limbs during prolonged standing, optimizes plantar pressure distribution, and maintains body stability. Future studies should use a more precise duration threshold of prolonged standing, better measurement of health outcomes, and more rigorous trial designs to develop a higher level of evidence to provide evidence-based recommendations and guidelines for reducing the health risks induced by prolonged standing.

## Figures and Tables

**Figure 1:** Schematic diagram of the sampling distribution.

**Figure 2:** The schematic diagram of the trial.

**Figure 3:** The photo of the testing site.

**Figure 4:** The schematic diagram of the plantar zones division (BH: hallux; OT: other toes; MF: medial foot; LF: lateral foot; M: midfoot; H: heel).

**Figure 5:** The plot of the sample size and statistical power.

**Figure 6:** Comparisons of perceived exertion and foot biomechanical parameters. (a) Perceived exertion. (b) COP amplitude. (c) Peak plantar pressure. (d) balance error scoring.

**Table 1:** Information of the eligible participants.

	Male	Female
Number	16	16
Age (year)	24.2 ± 1.8	23.6 ± 1.6
Height (cm)	178.6 ± 5.4	163.4 ± 4.2
Body weight (kg)	73.6 ± 5.2	57.3 ± 4.8
BMI (kg/m^2^)	22.9 ± 1.4	21.6 ± 1.7

BMI: body mass index.

**Table 2:** Comparison of perceived exertion and foot biomechanical parameters change within and between groups.

Items	Subitems	Group	Paired *t* test				Student's *t*-test	
			Before	After	Mean difference	*P* value	*T*	*P* value
RPE (point)	Foot	GS	0.96 ± 0.75	9.40 ± 0.71	8.43 ± 0.88	<0.05	2.60	<0.05
		MS	0.40 ± 0.49	8.20 ± 0.83	7.80 ± 0.87	<0.05		
	Shank	GS	0.90 ± 0.75	9.30 ± 0.74	8.40 ± 0.84	<0.05	2.95	<0.05
		MS	0.40 ± 0.49	8.13 ± 0.81	7.77 ± 0.76	<0.05		
	Knee	GS	0.97 ± 0.84	9.40 ± 0.71	8.43 ± 0.88	<0.05	2.95	<0.05
		MS	0.40 ± 0.49	8.10 ± 0.79	7.70 ± 0.69	<0.05		
	Thigh	GS	0.87 ± 0.85	9.30 ± 0.69	8.43 ± 0.84	<0.05	2.95	<0.05
		MS	0.33 ± 0.47	7.97 ± 0.71	7.63 ± 0.66	<0.05		
	Waist	GS	0.73 ± 0.73	9.33 ± 0.70	8.60 ± 0.10	<0.05	3.54	<0.01
		MS	0.33 ± 0.47	8.13 ± 0.72	7.80 ± 0.70	<0.05		
COP amplitude (mm)	X-axis	GS	1.51 ± 0.52	1.83 ± 0.48	0.32 ± 0.52	0.08	2.45	<0.05
		MS	1.77 ± 0.31	1.87 ± 0.32	0.10 ± 0.34	0.07		
	Y-axis	GS	11.58 ± 3.24	15.13 ± 4.56	3.55 ± 4.36	0.10	2.14	<0.05
		MS	12.90 ± 3.16	14.49 ± 3.67	1.59 ± 3.67	<0.05		
Peak plantar pressure (kPa)	BH	GS	5.95 ± 12.55	7.49 ± 13.71	1.55 ± 8.71	<0.05	0.56	0.581
		MS	9.20 ± 15.00	9.68 ± 13.64	0.48 ± 10.09	0.21		
	OT	GS	5.89 ± 11.65	10.49 ± 11.48	4.60 ± 9.95	<0.05	0.16	0.874
		MS	6.21 ± 9.73	11.29 ± 13.79	5.09 ± 9.55	<0.05		
	MF	GS	42.50 ± 18.80	53.16 ± 19.90	10.66 ± 22.26	<0.05	2.35	<0.05
		MS	35.50 ± 10.34	35.24 ± 11.97	−0.26 ± 9.05	0.46		
	LF	GS	70.11 ± 19.29	57.22 ± 18.53	−12.89 ± 15.24	<0.05	2.63	<0.05
		MS	47.78 ± 14.82	43.02 ± 10.36	−4.76 ± 11.68	0.14		
	M	GS	17.25 ± 12.81	29.90 ± 11.63	12.65 ± 13.70	0.25	2.60	<0.05
		MS	26.55 ± 9.27	29.76 ± 7.02	3.20 ± 6.14	0.30		
	H	GS	136.22 ± 22.46	147.77 ± 22.12	11.55 ± 16.32	0.44	2.95	<0.05
		MS	109.73 ± 29.20	111.48 ± 26.91	1.75 ± 7.78	0.55		
AI	AI	GS	0.15 ± 0.07	0.16 ± 0.06	0.06 ± 0.05	0.67	2.68	<0.05
		MS	0.15 ± 0.05	0.17 ± 0.04	0.02 ± 0.03	0.85		

GS: hard ground surface; MS: standing mat surface; BH: hallux; OT: other toes; MF: median foot; LF: lateral foot; M: midfoot; H heal; AI: arch index.

**Table 3:** Comparison of BESS score between groups.

Standing task	Difference between groups		*P* value
	GS	MS	
Standing on both feet (GS)	0.00 ± 0.00	0.00 ± 0.00	1.000
Standing on both feet (MS)	0.07 ± 0.26	0.14 ± 0.44	0.161
Standing on a single foot (GS)	2.07 ± 1.60	1.39 ± 1.70	0.011
Standing on single foot (MS)	2.32 ± 1.28	1.61 ± 1.78	0.014
Standing by lunge posture (GS)	1.36 ± 1.11	0.75 ± 0.87	0.048
Standing by lunge posture (MS)	1.89 ± 1.42	1.11 ± 1.80	0.023

GS: hard ground surface; MS: standing mat surface.

**Table 4:** Comparison of foot morphological change within and between groups.

Item	Group	Paired *t*-test within the group			Student's *t*-test between groups	
		Before	After	Mean difference	*T*	*P* value
Instep height(mm)	GS	74.70 ± 5.53	72.96 ± 4.70	−1.11 ± 7.23^∗^	0.004	0.997
	MS	74.50 ± 3.91	73.39 ± 3.76	−1.11 ± 6.16^∗^		
Ball of the foot length (mm)	GS	42.22 ± 8.04	41.02 ± 6.99	-1.02 ± 10.65^∗^	0.704	0.492
	MS	42.88 ± 4.65	41.54 ± 7.44	−1.34 ± 8.77^∗^		
AHI (%)	GS	30.00 ± 0.02	29.00 ± 0.01	−1.00 ± 0.02^∗^	3.540	0.003^∗∗^
	MS	32.00 ± 0.02	32.00 ± 0.02	0.00 ± 0.03		

GS: hard ground surface; MS: standing mat surface; ^∗∗^: *P* < 0.01; ^∗^: *P* < 0.05.

## Data Availability

Link: https://1drv.ms/u/s!Aqz2bCok6hp--y-ZM4Cg4E6fJB16?e=WoXoGJ.
